The article "Analysis of Mechanical Characteristics of Bionic Artificial Skin Using Different Suturing Patterns" was published in 2021. Journal: Appl Bionics Biomech.

# Analysis of Mechanical Characteristics of Bionic Artificial Skin Using Different Suturing Patterns

**DOI:** 10.1155/2021/6696612

**Published:** 2021-03-20

**Authors:** Tan Xiaohua, Xiao Xia, Li Qiu, Wang Lijie, Li Baizhou

**Affiliations:** ^1^Tianjin Key Lab of High Speed Cutting and Precision Machining, Tianjin University of Technology and Education, China 300222; ^2^School of Mechanical Engineering, Tianjin Polytechnic University, China 300387

## Abstract

Artificial bionic skin material is playing an increasingly important role in the field of medicine and bionic engineering and becoming a research hotspot in many disciplines in recent years. In this work, the digital moiré method was used to measure the mechanical field of the bionic skin material under different suturing conditions. Through the digital image process, the deformation characteristics and the stress distribution near the contact area between the bionic skin material and the suture were obtained and discussed. The different healing effects caused by suturing mode were further explored, which can provide mechanical guidance for wound suturing in clinical medicine.

## 1. Introduction

Artificial bionic skin materials are widely applied in the field of biology and clinical medicine. People can study the specific function of natural biological performance by simulating the natural biological structure using biomimetic skin material, which is essential in tissue engineering and regenerative medicine [1]. In clinical medicine and orthopedic surgery, the stress and deformation of skin tissue near the suture site are one of the direct factors impacting wound healing and scar formation; the surgeon in the operation needs to choose the way of suturing according to the shape and location of the wound [2].

Stress concentration usually occurs during the contact of the bionic skin material with the surgical suture. Hoy and Gingras [3] compared the effects of smooth suture and barbed suture on wound healing using photoelastic technique. Bucalo and Iriondo [4] used a transparent soft material similar to the earlobe tissue to simulate the suture of two different shapes of wound and observed the distribution of the stripes near the suture line through photoelastic measurement technology. John et al. [5] proposed a sensor for measuring the tensile deformation of a soft material, which utilizes the change in the reflectivity of the polarized light before and after the large deformation of the tissue and measured the stress changes of skin tissue before and after the surgical suturing. Yang et al. [6] evaluated the recovery of skin wounds after using three different suture treatments, including N, V, and NV shapes, taking into account the mechanical tensile strength and the effect of surgical line thickness [7]. At present, the study of wound healing is mainly based on histological analysis, lacking of considering mechanical factors.

Due to the characteristics of large deformation, Gao and Qian and Gao and Gao [8, 9] found that the deformation of soft materials can be divided into two configurations, that is, expansion and shrinking zone. This theory was validated by the experimental observations of Xia et al. [10]. Basing on the preliminary experimental work [10], this paper mainly focuses on the assessment of the displacement field, strain field, and stress distribution of skin wounds after using different suturing patterns. By studying the deformation law of the large deformation material under concentrated force, the mechanical characteristics of the area around the suture were obtained, and the influence of the suture on the wound recovery is discussed, which provides mechanical guidance for clinical surgery.

### 1.1. Digital Moiré Experiment of Bionic Skin

#### 1.1.1. Specimen Preparation and Experiment

Human skin tissue is nonuniform material, with nonlinearity, structure particularity, anisotropy, and specificity of physical and mechanical properties [11]. Mechanical properties of biological skin tissue are extremely complex, so the bionic material for human skin should have similar mechanical properties. The bionic skin material used in this paper was a kind of commercial soft matrix composite material (which was applied as the limb skin, provided by Tianyan Medical Science and Education Company). It is a special functional material with good flexibility. Before the experiment, the material was made into a rectangular specimen with a size of 15 × 4 mm for uniaxial tensile test. The thickness of the specimen was about 1 mm. The flow limit of the material was found to be 0.96 MPa, the Young modulus was 1.9 MPa, the maximum strength was 2.9 MPa, and the elongation was 520%.

The deformation fields of the area around the pinhole using I-shape and V-shape suturing pattern were measured by the digital moiré experiment method. The specimen shown in Figure 1(b) is an I-shape sutured specimen; the preparation process is as follows: firstly, the bionic skin material was cut into two 60 mm × 30 mm × 1 mm pieces; then, the two pieces of material were docked and stitched using a medical silk braided suture (Chinese traditional specification code: 1; diameter 0.2~0.249 mm), making sure the stitching edge of the area was directly contacted without fold and the surgical lines were straight. According to the suture standard of clinical surgery [12], the distance from the pinhole to the suture edge was 10 mm, the spacing between adjacent pinholes was 15 mm, and the suture length was 20 mm, which ensure the tensile direction was vertical to the wound.

Then, the black and white orthogonal gratings with a grid frequency of 3 dots/mm were prepared by spraying around the sutured area. Finally, the stitched specimens were fixed on the Instron 3343 electronic universal testing machine (load range 10 N~1000 N), applying a uniaxial tensile load of 2 mm/min. The experimental images were recorded by a BaslerA202K CCD camera (resolution 1003 pixel × 1004 pixel) and the associated image acquisition system. The second specimen was sutured using a V-shape pattern as shown in Figure 1(a) with a suture pitch of 7.5 mm and with the rest of the parameters the same as the previous specimen. Two samples of the deformed grating images of the two specimens are shown in Figure 1(c), respectively.

#### 1.1.2. Digital Moiré Process

In this paper, the orthogonal grating images captured at the load of 28 N are analyzed. The horizontal and vertical grid lines were extracted after image preprocessing, and then, the images were processed using digital moiré image technology, mainly achieved through GUI programming of Matlab software. The brief processes are shown in Figure 2.

The whole process can be divided into three steps. The first step is image preparation, in which the images of the deformed gratings were preprocessed and binarized, and the reference gratings were generated by the software. In this paper, the deformed grid lines were extracted into horizontal and vertical gratings, and then, a denoising was performed to enhance the gate line information. The collected images may be affected by the uneven illumination during the experiment. Therefore, the grating image was divided into several subregions, and the average gray value was selected as the threshold in each subregion. The second step is image processing. The binary transform grid diagram was superimposed on the four phase shift reference grid graphs, and the logical moiré pattern was obtained by logical operation. Wavelet decomposition was applied to the logical moiré image, and the high-frequency noise was filtered by selecting a proper threshold. And then, a clear, continuous digital moiré pattern was obtained after fringe reconstruction using low-frequency information. After the parcelled phase diagram was calculated, the Macy algorithm was used to get the unpacked phase diagram. The phase map without wrapping corresponds linearly to the fringe series distribution. Given the phase value of the fringe order zero, the phase value of each point can be determined, and then, the displacement map of the whole field was obtained. Finally, a data file was generated from the resulting deformation distribution information.

### 1.2. Result Analysis

#### 1.2.1. Displacement Pattern

After the digital image processing, the displacement field information in vicinity of the suture area was directly obtained. By coordinate transformation, the displacement fields are presented in radial and circumferential form for better illustrating, as shown in Figure 3. In the figure, the pinhole of the suture was set as the origin of the coordinate, where the nearby material deformation was complicated. The pinhole area is marked out by circular dotted lines in Figure 3.

It can be seen from the displacement field information that the bionic skin material clearly exhibits the characteristics of the section configuration near the area in contact with the suture. If set *u*_*r*_ ≈ 0 as characteristic lines (i.e., the black dotted line in the figure), the observation area can be divided into two different regions. In Figure 3(a), the four characteristic lines divide the deformation field into four fan-shaped regions; the displacement of the upper and lower sectors is negative; that is, the particles were moving towards the origin, and the left and right sectors are positive, suggesting particles moving away from the origin. In Figure 3(b), the characteristic lines composed by *u*_*θ*_ ≈ 0 (gray dashed lines) are approximately located near the center of the four sectors. The characteristics of the displacement field show that after loading, the upper and lower sectors are the expansion zone, where the material approaches the concentrated force acting point in the radial direction, and become wide and occupy the majority of the sharp angle area, marked as EX in Figure 3; the left and right sectors are shrinking zones in which the material is radially detached from the pinhole area and contracted in the circumferential direction. This section becomes narrow and occupies only the smaller corner area after deformation, marked as SH in Figure 3.

It can be found that the partitioning features of the expansion zone and shrinking zone can be found near the pinhole both in I-shape and V-shape sutured specimens. The difference is that the displacement field of I-shape suturing is composed of four sectors, and the fan-shape area of the V-shape suturing is composed of three parts. The possible reason for the difference is that, under the same load, the specimens were subjected to equivalent concentrate forces in the vertical direction, the component force in the horizontal direction will cause the shrinkage zone of the second specimen under the action of the V-concentrated force, and the range of the shrinkage zone is related to the angle of the suture lines. Due to this reason, the expansion deformation on top of the suture point was weakened or offset.

#### 1.2.2. Strain Fields

To understand the rule of sector division more intuitively, the experimental results were transformed into the strain field under the polar coordinate system, using the displacement-strain relation shown in Equation (1).

(1) $$\begin{array}{c} \left.\begin{array}{c} \varepsilon_{r}=\frac{\partial u_{r}}{\partial r}+\frac{1}{2}\left[{\left(\frac{\partial u_{r}}{\partial r}\right)}^{2}+{\left(\frac{\partial u_{\theta }}{\partial r}\right)}^{2}\right],\\ \varepsilon_{\theta }=\frac{1}{r}\frac{\partial u_{\theta }}{\partial \theta }+\frac{u_{r}}{r}+\frac{1}{2}\left[{\left(\frac{1}{r}\frac{\partial u_{\theta }}{\partial \theta }+\frac{u_{r}}{r}\right)}^{2}+{\left(\frac{1}{r}\frac{\partial u_{r}}{\partial \theta }-\frac{u_{\theta }}{r}\right)}^{2}\right],\\ 2\varepsilon_{r\theta }=\frac{\partial u_{\theta }}{\partial r}+\frac{1}{r}\frac{\partial u_{r}}{\partial \theta }-\frac{u_{\theta }}{r}+\frac{\partial u_{r}}{\partial r}\left(\frac{1}{r}\frac{\partial u_{r}}{\partial \theta }-\frac{u_{\theta }}{r}\right)+\frac{\partial u_{\theta }}{\partial r}\left(\frac{1}{r}\frac{\partial u_{\theta }}{\partial \theta }+\frac{u_{r}}{r}\right), \end{array}\right\}, \end{array}$$

where *∂u*_*r*_/*∂r*, *∂u*_*r*_/*∂θ*, *∂u*_*θ*_/*∂r*, and *∂u*_*θ*_/*∂θ* are the partial derivatives of the displacement components in the polar coordinate system. The strain field at each point can be directly calculated from the displacement by interpolation. Since the strain is a secondary information, errors are inevitable in this process, the noise of the displacement field was filtered out by wavelet transform in this work, and then, the strain field was calculated based on the large deformation theory. The radial strain field *ε*_*r*_, the circumferential strain field *ε*_*θ*_, and the shear strain field *ε*_*rθ*_ of the pin tip region are shown in Figure 4.

The cool color in the figure represents a negative value, and the warm color represents a positive value. It can be seen that the radial strain is negative and the circumferential strain is positive in the upper region of the suture point, and the shear strain on the left and right sides of the surgical line is opposite. These features indicate that the material in this region produces radial compression and annular expansion under the extrusion of the surgical line. The material deforms towards the suture point in the radial direction and extends around the suture point in the circumferential direction. The radial strain is positive, and the circumferential strain is negative in the lower position of the concentrated force point. The shear strains on the left and right sides of the surgical line are also opposite, indicating radial stretching and circumferential shrinkage in this area, which is just opposite to the deformation in the upper area of the suture point. In conjunction with the displacement field results, it can be seen that the displacement and strain values are almost zero in the area surrounded by the two intersecting sutures, indicating that the deformation of the region is relatively small and remains relatively stable under external loads.

It can be seen that the bionic skin exhibits a sector division configuration of expanding sector and shrinking sector under the tension of I-shape and V-shape sutures. However, differences can be seen in the two cases after comparison. There are four fan-shape zones under the action of I-shape suturing, and only three sectors can be found in the V-shape suturing. In the latter case, there is a triangular region within the range of the intersection of the surgical lines, where the strain is gentler and the circumferential strain is slightly contracted. The difference in the configuration of the two suture patterns will affect the healing of the wound to a certain extent.

### 1.3. FEM Analysis

By inputting the experimentally measured mechanical properties of bionic skin materials into ABAQUS software, finite element analysis was performed to further explore the effect of suturing on wound healing. The constitutive model and its parameters were optimized by a variety of fitting methods. And then, numerical models were established on this basis. The geometrical and material parameters of the numerical models were the same as those of the experiment. The image with the external load of 28 N was analyzed. The distributions of the principal stress are shown in Figure 5.

It can be seen from the figure that the differences of the distribution of the principal stress between the two cases are not very evident. The values are apparently different. In the relevant medical analysis, the “average stress index” (ASI), i.e., the ratio of the principal stress integral to the area in the calculated area, is commonly used to assess the stress level near the suture [13]. In this paper, the principal stress values near the suture area are extracted from the finite element analysis results and the ASI near the pinhole was calculated. The results are shown in Table 1. It can be seen that the ASI produced by the V-shape suturing is larger than the I-shape suturing. This can provide useful clinical information for the surgeon since stress is an important factor in the healing of the wound.

## 2. Discussion and Conclusions

In the above two experiments, the incision of bionic skin can remain fixed under the constraints of the surgical suture and showed a similar deformation law. Deformation differences can also be found according to the displacement and strain field, which will have some effect on the recovery of the wound. In the case of I-shape suturing, the expanding sector appears on both sides of the surgical line, and the material in this region is moving towards the contact point and extends towards both sides with the suture as the center. In the V-shape suturing case, little movement can be seen in the triangular region surrounded by the suture intersects due to the restriction of the suture.

When held under tension, an expansion sector that deviates from the edge of the wound and caused by the vertical concentrate force (I-shape suturing) appeared near the contact area. This is not conducive to the recovery of the wound and may lead to scars after cure. The deformation of the wound is relatively much smaller in the triangular area surrounded by surgical sutures under the action of crossconcentrated force (V-shape suturing), indicating that the V-shape suturing can play a more stable role in the wound healing under the same external force. Moreover, the concentrated stress can be dispersed by V-shape sutures, resulting in a wider area of expanding sector with smaller strain gradient, which is a positive factor for wound recovery. Selecting an appropriate suture density can further reduce the strain gradient, hence promoting wound recovery.

In addition, the value of ASI is greater in V-shape suturing than I-shape suturing. Sutures can provide appropriate mechanical support during the wound healing period, but the relevant local stress caused by the sutures also can change the wound repair environment to a certain extent. Wound healing is a complex process where moderate stress can stimulate growth factors conducive to wound healing. However, excessive stress can cause wound inflammation, cracking, ischemia, and even gangrene phenomenon, because transitional restrictions on the deformation of the wound, especially in the triangle area surrounded by crossed sutures, will lead to local poor blood circulation and subcutaneous nervous system obstruction, leaving the drug and nutrition cannot be normally delivered to the wound, affecting tissue regeneration and repair. In addition, material instability phenomenon may happen when the stress level reaches or exceeds a certain threshold, resulting in surface wrinkles affecting the appearance.

Based on the above analysis, it can be seen that the suturing pattern can affect the level and mode of constraint near the wound area even under the same external force. Therefore, the appropriate suturing pattern should be chosen according to the following situations: V-shape suture can effectively promote wound healing in common cases; but for joints with more frequent movement or patients with skin microcirculation disorders, I-shape suturing is more suitable. In addition, skin wrinkles may easily caused by large stress concentration, which will affect the appearance of the human face skin. However, it can also promote nutrient absorption in the esophagus, intestine, and other parts of the wall mucosa, playing an important physiological role. Hence, this factor also needs to be considered in the choice of suture pattern. V-shape suturing should be recommended for the skin, and the I-shape suturing is recommended for inner lumen structures.

It is worth mentioning that this article mainly focuses on the effects of stress and deformation on wound healing, but the wound healing of real skin is a complex process. In addition to mechanical stimulation, the motion state, nutrition intake, drug delivery, surgical technique, radiation, cytokines, and other complex physical and chemical factors can also have great influence. The authors are currently preparing an animal skin suture experiment to conduct a comprehensive consideration.

## Figures and Tables

**Figure 1:** Experimental measurement of large deformation bionic skin using V-shape suturing (a) and I-shape suturing (b), respectively. Unit of lengths: mm.

**Figure 2:** Flow chart of digital image processing.

**Figure 3:** Displacement fields near the pinhole area of tensile bionic skin: (a) radial displacement of I-shape suturing; (b) circumferential displacement of I-shape suturing; (c) radial displacement of V-shape suturing; (d) circumferential displacement of V-shape suturing. Units: mm.

**Figure 4:** Strain fields of bionic skin under polar coordinate system. Units: %.

**Figure 5:** Distribution of principal stress near the pinhole of bionic skin, I-shape (a) and V-shape (b) suturing. Units: MPa.

**Table 1:** The average stress index (ASI) of bionic skin in an area of 19 × 19 mm^2^.

	Principal stress *σ*_1__(GPa)_	Principal stress *σ*_3__(GPa)_
I-shape suturing	0.067	-0.262
V-shape suturing	0.081	-0.282

## Data Availability

All the underlying data can be found through the authors. Anybody who is interested in the data can email the authors directly.
